This article has been retracted.

# The Acceptability of Traditional Culture under the Background of Deep Learning

**DOI:** 10.1155/2022/4010099

**Published:** 2022-08-23

**Authors:** Qian Sima, Shan Wu

**Affiliations:** ^1^School of Fine Art and Design, Kunming University, Kunming 650214, Yunnan, China; ^2^School of Information Management and Engineering, Shanghai University of Finance and Economics, Shanghai 200433, China

## Abstract

The cultural values of a country impact its national psychology and identity. Citizens' values and public opinions are conveyed to state leaders over the media and other information channels, both directly and indirectly influencing decisions on foreign policy. The traditional cultural values that affect the psyche of the Chinese people are harmony, generosity, morality, courtesy, wisdom, honesty, loyalty, and filial piety. This study aims to analyze the attitudes of Chinese college students toward traditional culture. The reliability and effect factors of the traditional culture acceptability questionnaire are set in the context of deep learning. A questionnaire on traditional culture education of college students is compiled using the indicator evaluation methods, and the current situation of traditional culture education is investigated for college students. A total of 300 valid respondents are returned from five universities including Shanghai Jiaotong University, Fudan University, Yunnan University, Kunming University of Science and Technology, and Yunnan Normal University. Results show that 28% of college students believe that practical activities including visiting and learning and traditional festival commemoration are the most effective ways to educate traditional culture for them, which accounts for the largest percentage. Similarly, 19% of students suggest online publicity, while 16% believe that lecture reports are particularly important, and 12% of students advocate the teaching courses. In addition, about 23% of the students choose other methods, such as seminars, setting up Chinese culture festivals, and building cultural associations. The outcomes of this study provide data support for identifying the shortcomings in traditional cultural education and formulating strategies.

## 1. Introduction

For a country and a nation, culture is the guarantee for survival and is a symbol that distinguishes it from other countries and nations [1]. Since the 40 years of reform and opening up, the development of China has attracted worldwide attention and made excellent achievements [2]. However, China's cultural field has been eroded and even impacted by multiculturalism from all over the world while achieving leapfrog development in the fields of politics, economy, and military. The cultures of various countries have gradually entered China, and there are sparks and conflicts with the Chinese culture. Some Western countries even use cultural exchanges as a powerful means to import their cultural values into China, which has seriously threatened Chinese traditional culture. In the context of this era, China has to take the improvement and enrichment of national traditional cultural education as the primary task for construction [3].

The investigation of traditional culture all over the country has enriched the research in the field of culture. Huang et al. [4] believed that the economic and social effects of traditional Chinese culture affect the measurement of culture. Guo [5] proposed that in the face of the impact and influence of foreign cultures, the expansion of traditional culture is threatened, so it has to strengthen the protection and inheritance of traditional culture. Yang et al. [6] considered that China is an ancient civilization with history and culture of 5,000 years and has inherited many excellent traditional cultures. Recently, China has begun to attach importance to the protection and inheritance of traditional culture, and explore the integration of traditional culture into the teaching of various disciplines. However, there are still problems such as low degree of integration and formalized teaching in the process of integrating specific disciplines and maker education courses. Htet and Leslie [7] argued that the questionnaire ordinal scale asks respondents how much they agree with a given statement and adopted the multiple linear regression analysis methods to measure the degree of influence of cultural invasion on traditional culture to protect its ancestral culture. In the field of deep learning, Shorten et al. [8] evaluated the current state of deep learning for natural language processing for information retrieval and question answering, as well as misinformation detection and public sentiment analysis. Dong [9] introduced the structural principles, characteristics, and several classical models of deep learning, such as stacked autoencoders, deep belief networks, deep Boltzmann machines, and convolutional neural networks. Ranganathan [10] surveyed recent advances in the application of modern computer vision techniques (driven by deep learning) to traditional culture and briefly summarized the ten-year progress of convolutional neural networks, including their visual manifestations in traditional cultural contexts. Liu [11] discussed the current situation and problems of the acceptance status of excellent traditional moral culture among college students and analyzed the aspects that limit the receipt of excellent traditional moral culture among college students to complete a large-scale analysis on the acceptance status of traditional moral culture in colleges and universities. A model based on convolutional neural networks is proposed for predicting college students' acceptance of traditional moral values. By learning and describing their activities and preferences on the Internet, the model evaluates and creates college students' acceptance status for conventional moral culture. The author in [12] suggested that colleges and universities should make extensive use of social media to encourage the formation of traditional moral culture among students and it gives college students a suitable teaching platform for traditional moral culture instruction.

In this study, the attitudes of Chinese college students toward traditional culture are analyzed. The reliability and effect factors of the traditional culture acceptability questionnaire are set in the context of deep learning, and the Questionnaire on Traditional Culture Education of College Students is compiled using the indicator evaluation methods given in the traditional culture acceptability questionnaire. Results show that most college students think that practical activities are effective to teach traditional culture in colleges and universities. A small number of students suggest the method of online publicity, and the rest believe that other methods are effective means, such as exchange seminars, setting up Chinese culture festivals for college students, and building cultural associations. The survey results provide data support and practical significance for the development of traditional cultural education.

The rest of the manuscript is organized as follows: Section 2 is data collections and methods.  Section 3 illustrates different results for analysis on survey of the traditional culture acceptability questionnaire, and the conclusion is presented in Section 4.

## 2. Methods

### 2.1. Setting the Reliability and Effect Factors of the Traditional Culture Acceptability Questionnaire

The process to set the reliability and effect factors of the traditional culture acceptability questionnaire is given in Figure 1.

The following three points are taken into account while considering the reliability coefficient.

- In different situations, different reliability coefficients can be obtained for different sample data by using different methods, so a test may have more than one reliability coefficient.
- The reliability coefficient is only an estimate of the degree of inconsistency of the measurement scores and does not point out the reasons for the inconsistency.
- Obtaining a higher reliability coefficient is not the ultimate goal of the measurement, but is only a step toward the goal, which is a necessary condition for the test to be effective.

If the reliability coefficient is used to represent the size of the reliability, the larger the reliability coefficient, the greater the reliability of the measurement [13]. However, existing similar tests can be used as a benchmark for comparison. For the ability and achievement test, the measured *y*_*xx*_ should be greater than 0.91 to ensure validity, and a questionnaire with a *y*_*xx*_ of 0.95 can be regarded as an excellent questionnaire. For personality tests such as personality, interests, and values, it is more appropriate for the measured *y*_*xx*_ to be greater than 0.80 and less than 0.85, and it can be appropriately larger. If *y*_*xx*_ is less than 0.70, then the questionnaire is not suitable for individual evaluation, nor is it suitable for comparison between groups. For group comparison, *y*_*xx*_ should be greater than or equal to 0.70, while it should be greater than or equal to 0.85 to identify individuals [14].

If *X* is defined to represent the actual score (observed score) measured by the questionnaire, then the actual score can be computed as

(1) $$\begin{array}{c} X=T+B+E, \end{array}$$

where *B* is the systematic error (deviation score) of the questionnaire and *E* refers to the random error (measurement error). True dispersion is an abstract concept or a potential variable. The observed values *X* and *T* obtained in the actual measurement may not be completely consistent [12]. For the measurement error, it is generally assumed that its expected value is 0, and it is independent of the true score [13].

Under this assumption, it can be concluded that the mean of the actual scores and the measured scores is generally equal and can be expressed using (2) and (3), respectively.

(2) $$\begin{array}{c} E\left(X\right)=E\left(T\right), \end{array}$$

(3) $$\begin{array}{c} \sigma_{x}^{2}=\sigma_{t}^{2}+\sigma_{e}^{2}, \end{array}$$

where *E*(*X*) and *E*(*T*) are the expectations of measured *X* and predicted *T*, respectively. The variance *σ*_*x*_^2^ of the measured score is equal to the sum of the variance *σ*_*t*_^2^ of the true score and the variance of the error *σ*_*e*_^2^. The ratio of the variance of the general true score to the total variance is called reliability [15], which can be expressed as follows:

(4) $$\begin{array}{c} y_{xx}=\frac{\sigma_{t}^{2}}{\sigma_{x}^{2}\left(1-\sigma_{e}^{2}/\sigma_{x}^{2}\right)}. \end{array}$$

Or the reliability can be defined as follows:

(5) $$\begin{array}{c} y_{xx}=\sqrt{\frac{\sigma_{t}^{2}}{\sigma_{x}^{2}}}, \end{array}$$

where *σ*_*x*_^2^ is the variance of *x*, *σ*_*t*_^2^ is the variance of the true score, and *σ*_*e*_^2^ refers to the error. (4) expresses the reliability as a form of a correlation coefficient, which is realized by the correlation between the true score and the measured score [16]. In (5), the reliability is expressed as the ratio of the variation between the actual traditional culture respondents' questionnaire scores and the predicted values, which is the square of the correlation coefficient, or as the difference between the traditional culture respondents' questionnaire scores and the predicted scores coefficient of determination. It is very similar to the coefficient of determination introduced in the one-way analysis of variance (ANOVA) for regression [17]. Most of the reliability indicators are represented by the correlation coefficient, which is called the reliability coefficient, indicating the correlation between the two groups of data obtained from the same sample is used as an indicator for measuring consistency [18].

Validity is related to the purpose of measurement. The same measurement tool has high validity in some measurements, but not in others [19]. For example, a ruler with high reliability has good validity in measuring height, but not in measuring blood pressure. Therefore, validity can also be defined as the degree to which a test can achieve a certain purpose [20].

### 2.2. Construction of Indicator System in the Traditional Culture Acceptability Questionnaire

The indicator system is not a simple collection of multiple indicators, but an organic whole formed by multiple indicators. The construction of the indicator system structure is shown in Figure 2.

The indicators of the traditional culture acceptability questionnaire should follow the following principles.

- Scientific: Each indicator of the questionnaire should have a certain scientific connotation, and the indicators of the questionnaire system should be determined according to the effective utilization of the data obtained by the questionnaire, reasonability of obtained data, and the relevant design principles of the questionnaire.
- Integrated: Sufficient and complete information should be used to support the evaluation objectives in the indicator evaluation system, so that the evaluation conclusion is fair, guaranteeing the effectiveness of the index system [21].
- Purposive: The purpose of constructing the indicator system is to evaluate certain situations, so it is necessary to clarify one's own goals to construct an indicator system; otherwise, the indicator system will not exist.
- Clear structure: The hierarchy of the indicator system should be clear, and the analysis and summary should be convenient.
- Systematic.
- Operable: The data of a single indicator that is desirable and easy to calculate should be selected, and the operability of the calculation of the indicator directly affects the effectiveness of the indicator system.
- Dynamic: Things are constantly developing and changing, so the corresponding design of the indicator system should maintain certain flexibility, to modify and update them according to new conditions and situations.
- Independent: The evaluation results should be reliable and accurate. The mutual independence of each indicator and the indicator system should be scientific and reasonable.

### 2.3. Indicator Evaluation Method in the Traditional Culture Acceptability Questionnaire

In the traditional culture acceptability questionnaire, the response rate of respondents is the top priority, which is related to the smooth progress of the survey and the accuracy of the experiment. It can be represented as

(6) $$\begin{array}{c} F=\frac{V}{T}, \end{array}$$

where *F* represents the response rate, *V* shows the number of valid questionnaires recovered (where the valid definition is consistent responses before and after, and the experience of filling out the questionnaire), and *T* refers to the total number of questionnaires issued. In the survey data, *T* is to record the total number of distributions, which means that the *T* variable is increased by 1 for each distribution, then another variable *V* is adopted to record the number of replies received, and each time a reply questionnaire is received, the *V* variable is also automatically increased by 1. After the invalid questionnaires, such as questionnaires that did not answer all the questions, are manually eliminated, the response rate at this time is the ratio of the two variables *T* and *V* [22, 23].

The difference is another important parameter in the questionnaire which can be computed as follows:

(7) $$\begin{array}{c} D=\min\left\{\frac{X_{1}}{X},\frac{X_{2}}{X},\cdots ,\frac{X_{n}}{X}\right\},\\ T=\max\left\{\frac{X_{1}}{X},\frac{X_{2}}{X},\cdots ,\frac{X_{n}}{X}\right\}, \end{array}$$

where *X*_*n*_ represents the number of people who choose the n^th^ group of options, *X* refers to the total number of people, the minimum degree of difference is *D,* and the maximum degree of difference is *T*. The specific calculation steps of difference are summarized as follows. (i) It should calculate *D* and *T* first. (ii) If *D* is less than 3% or *T* is greater than 70%, it means that the option design is unreasonable and has to be modified. On the contrary, it means that the options of the questionnaire are quite different, which can reflect the different situations of most people [24].

In the split-half reliability analysis, important content is to evaluate the degree of correlation between the two scales. The main purpose is to analyze the common questions asked by the two-part scale. When the external reliability is analyzed, if it needs to judge the conceptual ambiguity and ambiguity, it has to analyze the correlation between the two evaluation results. When the internal reliability is analyzed, a reliability study is mainly carried out, which is the reliability level of only half of the project evaluation [23]. The specific steps are as follows:

- The total score of each evaluated object on the two-part evaluation items is calculated.
- The simple correlation coefficient of the total score is computed and is denoted as *R*_*XX*_.
- *k* is biased under certain circumstances. It means that when there are not many evaluation items, they should be corrected. If the number of evaluation items in the two parts is equal, the Spearman–Brown correction method [24] is adopted and is expressed as follows:

(8) $$\begin{array}{c} R_{XX}=\frac{2R_{XX}}{1+R_{XX}}, \end{array}$$

where *R*_*XX*_ is the simple correlation coefficient of the total score. If the number of evaluation items in the two parts is inconsistent, then the definition of *R*_*XX*_ should be as follows from the perspective of variance:

(9) $$\begin{array}{c} R_{XX}=2\left(1-\frac{S_{1}^{2}+S_{1}^{2}}{S^{2}}\right), \end{array}$$

where *S*^2^ is the total variance of the two parts, *S*_1_^2^ is the variance of the total score of the first part, and *S*_2_^2^ shows the variance of the total score of the second part [25]. The split-half reliability method refers to the consistency of the scores measured by the two half-scales, and the corona coefficient represents the consistency between the scores of each item on the scale. What they analyze is the consistency within the scale. If there is no correlation between the item in the scale and one of the items, it means that the scale does not contain this item, and this item needs to be eliminated. Reliability analysis can be carried out on any questionnaire, and the specific evidence of the goodness of the test and scale is the objective indicators provided [26–28]. The reliability value can be judged with the below equation.

(10) $$\begin{array}{c} \theta =\frac{k}{k-1}*\left(1-\sum \frac{S_{1}^{2}}{S_{x}^{2}}\right), \end{array}$$

where *k* represents the number of parameters in the breakdown. ∑*S*_1_^2^ is the variation of scores (*I* = 1, 2,…, *k*) for all respondents when the item *i* is optional, and *S*_*x*_^2^ refers to the variance of the total score of all respondents. The sum of the points scored by respondents in each item is their total score. If there are enough items and the coefficient *a* is low, it means that some items are not of one type and have to be eliminated.

## 3. Results Analysis

### 3.1. The Selection of the Questionnaire Sample and the Respondents' Tendency toward Chinese Classics

In this study, the students of Shanghai and Yunnan colleges are taken as the survey objects, and paper questionnaires and online questionnaire promotion are adopted to achieve random sampling and scientific accuracy of the questionnaires. To excavate the inheritance of traditional culture by undergraduates in the country from a deep level, it can explore the attitudes of college students toward the traditional culture from the perspective of undergraduates' learning and behavioral status and the objective evaluation of traditional culture to explore the necessity and feasibility of self-confidence education in colleges and universities. The specific survey objects are shown in Figure 3.

The subjects of the online questionnaire survey are college students from Yunnan University, Kunming University of Science and Technology, and Yunnan Normal University, which are surveyed using a completely random sampling method. The respondents of the paper questionnaire are the college students of Shanghai Jiaotong University and Fudan University, where the method of cluster sampling is adopted. A total of 300 valid questionnaires are collected through two methods, including 169 students majoring in humanities and social sciences, 61 students majoring in science and medicine, and 70 students majoring in arts and sports. There are 65 freshmen, 79 sophomores, 89 juniors, 67 seniors, and 4 who have graduated. There are 153 males, accounting for about 51%, and 147 females, accounting for about 49%. The proportion of male and female respondents is average, and the sample selection is relatively reasonable.

For literary classics such as Mencius, “The Doctrine of the Mean,” “The Book of Songs,” and “The Spring and Autumn Period,” the reading intentions of college students are shown in Figure 4.

Figure 4 illustrates the attitude of current college students toward classic sinology. Among the total students, 45 students are not willing to read Chinese classics, accounting for about 15% of the total, and they should strengthen the influence of traditional culture. There are 34 students who are indifferent to sinology, accounting for 11%, and they should pay attention to the reading of sinology. Fortunately, the remaining 221 students have read classic sinology or are very interested in sinology, accounting for 74%, of which 23% expressed a strong interest in reading sinology, which is the backbone of the country. In the gender dimension, compared with male groups, female students are significantly more interested in sinology than male students. To sum up, we should not hold pessimistic prospects for the reading of Chinese classics by college students. Most groups are willing to read, and for a small group, the cultivation of their Chinese literacy should be strengthened.

### 3.2. The State of College Students' Cultural Courses and the Differences between Chinese and Western Cultures

Cultural courses are one of the few traditional cultural education courses that can be contacted by students during the university period. For the study of cultural courses for college students, this topic is based on multiple-choice questions. The specific status is shown in Figure 5.

As revealed in Figure 5, 300 college students in the sample answer a total of 622 choices, with an average of about 2 choices per person. Among these options, 232 people chose “Chinese traditional excellent cultural courses,” accounting for 37%, followed by “socialist reform and development courses” selected by 156 students (accounting for 25%). It seems that with the call of the party and the country, college students are paying more and more attention to China's development. But there are also a large number of students who choose Western culture courses including 132 students, accounting for 21%. It can be known that Western culture is slightly changing the thinking of college students. The least selected are the red cultural courses and other cultural courses, both of which are less than 10% of the total. This shows that college students should cultivate their study of red culture courses.

With the advancement of globalization, the integration of Chinese and Western cultures has become deeper and deeper. In this questionnaire, the degree of influence of Chinese and Western cultures on college students is very important. The specific data are shown in Figure 6.

In terms of the impact of Chinese and Western cultures on college students, 221 college students believe that both Chinese and Western cultures have a greater impact on themselves. Among them, 185 respondents favor that Chinese culture has a greater influence on themselves, accounting for about 62%, of which 119 are boys and 666 are girls. Only 21 students are loyal to Western culture, accounting for less than 10%. The number of people who love Chinese culture is 56, including 31 boys and 16 girls. This indicates that in the struggle between Chinese and Western cultures, the students' acceptance of Chinese culture is still very high at this stage. However, there is also a small number of groups that are deeply influenced by Western culture, among which women are more than men. It seems that women are still more deeply poisoned by consumerism and hedonism in the trend of thinking in Western culture.

### 3.3. Analysis of College Students' Acceptability of Traditional Culture Channels and Chinese Culture Inheritance

At the current stage of university education, it is necessary to master the channels through which college students receive traditional culture. The different channels are shown in Figure 7.

In terms of channels for college students to receive traditional culture, books and magazines are the main ways for college students to acquire traditional culture, which is selected by 89 students (accounting for about 30%), including 43 boys and 46 girls. The second is the situation policy course, the campus network, and the general education course, all of which account for about 20%. However, only 4 students acquire culture in other ways, which is less than 2%. This confirms college students are diverse in the acquisition of traditional culture.

In the modern age where traditional Chinese culture is gradually declining, it is necessary to investigate the reasons for its decline. The reasons for the cultural decline are shown in Figure 8.

Figure 8 reveals that 98 respondents believe that the reason for the cultural decline is the comprehensive suppression of traditional culture after the May 4^th^ Movement, and the overall westernization, accounting for 33%. There are 65 respondents that believe that it is the invasion of Western culture, occupying the Chinese market, such as Hollywood blockbusters in the USA and comics by Ruben. Hedonic and money-worshiping in the market economy also have a greater impact on young people, and the number of people who maintain this argument is 78, accounting for 26%. However, the number of students who maintain the view of cultural faults and lack of government protection of traditional culture is relatively small, only 7% of the population.

### 3.4. Socialist Values and the Problems of University Traditional Culture Education

Since the 19^th^ National Congress of the Communist Party of China, the mastery of the socialist core value system has been deeply rooted in the hearts of the people. The socialist core values are the main body of the value system, and college students are also the main body of the masses. The educational situation of socialist core values is shown in Figure 9.

As the results are shown in Figure 9, the frequency of 218 students participating in the education of socialist core values is multiple times, accounting for about 73%. Such a result is very gratifying. There are 67 students who participate occasionally, accounting for about 23%, and they need to strengthen political education. Another 15 respondents express no interest in the education of socialist core values. From the perspective of gender ratio, the ratio of males and females is even, whether it is a strong will or lack of interest in the education of socialist core values.

There are more or less such problems in the process of university traditional culture education. In response to this problem, the views of the students are shown in Figure 10.

It can be known that 15.3% of the students believe that the problem in the process of traditional and ancient culture education in new era universities is that the cultivation method is too single, and the opinions of male and female students are roughly the same. Among them, 29% of college students believe that in the process of traditional cultural education in universities in the new era, the enthusiasm of students is insufficient, and there are more boys than girls who hold this view. Similarly, 26.3% of the college students believe that in the process of self-confidence education of traditional culture in the new era, publicity and guidance are superficial, and there are far more girls than boys in this view. There are also 29% of college students who believe that in the process of traditional cultural education in universities in the new era, the school does not pay much attention to it, and there are slightly more boys than girls. In a word, the above four types of problems are common in the process of traditional cultural education in universities in the new era.

### 3.5. Optimization of Traditional Culture Education in Universities

Given the problems in the traditional culture education in universities, effective measures should be taken. The measures proposed are shown in Figure 11.

These options in Figure 11 demonstrate that 28% of college students choose practical activities (visiting and learning, traditional festival commemoration, etc.) as an effective way of university traditional culture education, which is the largest proportion. Second, 19% of students suggest online publicity, while 16% of students believe that lecture reports are particularly important, and 12% of students advocate the establishment of courses as an effective way to educate traditional culture in universities. About 23% of the students choose other methods, such as exchange seminars, setting up Chinese culture festivals for college students, and building cultural associations.

## 4. Conclusion

Investigation of the educational methods of traditional culture in universities and colleges reveals that traditional education channels such as humanities general courses, ideological and political courses, books, newspapers, and magazines are the main sources for college students to receive traditional education. In this study, the attitudes and tendencies of Chinese college students toward traditional culture were analyzed. A questionnaire on traditional culture education of college students was compiled using the indicator evaluation methods. A total of 300 valid respondents were returned from five Chinese universities. It is also found that college students generally believe that practical activities are the most effective way of the traditional culture education and practical activities in the form of visiting and learning and celebrating traditional cultural festivals can mobilize the enthusiasm of students to actively participate. Moreover, the construction of cultural associations, the establishment of special Chinese culture festivals for college students, and the establishment of related courses are all considered to be better educational methods. In addition, carrying out traditional cultural education in a form that college students are willing to accept will surely achieve better educational results. Regarding the implementation status of traditional culture education in universities, universities should let college students have more understanding of traditional culture, to inspire them to actively participate in traditional culture education activities and achieve the expected results of traditional culture education. Although the outcomes of this analysis are promising, the results of this study are based on the students of only five Chinese universities. Further investigation is required to large number of students from other Chinese universities.

## Figures and Tables

**Figure 1:** Process of setting the reliability and effect factors of the traditional culture acceptability questionnaire.

**Figure 2:** The construction of the indicator system in the traditional culture acceptability questionnaire.

**Figure 3:** The selection of the questionnaire sample of the traditional culture acceptability questionnaire.

**Figure 4:** The willingness tendency of college students to the Chinese classics.

**Figure 5:** The study status of college students' cultural courses.

**Figure 6:** Differences in the influence of Chinese and Western cultures on college students.

**Figure 7:** Channels for college students to receive traditional culture.

**Figure 8:** Analysis of factors affecting the inheritance of Chinese culture.

**Figure 9:** Educational situation perception of socialist core values.

**Figure 10:** Problems in traditional culture education in universities.

**Figure 11:** Optimization of traditional culture education.

## Data Availability

The data used to support the findings of this study are available from the corresponding author upon request.
